The article "Big Data Analysis of Benign Interaction of Great Power Relations and New International Relations Based on Deep Learning" was retracted in 2023. Reasons: signs of a paper mill; suspected computer-generated content; unreliable results or conclusions; lack of ethics approval or compliance.

# Big Data Analysis of Benign Interaction of Great Power Relations and New International Relations Based on Deep Learning

**DOI:** 10.1155/2022/9714591

**Published:** 2022-08-22

**Authors:** Yanhong Ma

**Affiliations:** School of Politics and International Relations, Tongji University, Shanghai 200000, China

## Abstract

The development of a new type of international relations is the advancement and improvement of diplomatic thinking among contemporary nations. It also serves as a crucial yardstick for assessing the future global pattern and the direction of order changes. Proper interaction between major powers can foster the growth of new international relations and has a significant impact on advancing global cooperation and the promotion of human peace. The goal of this essay is to examine how friendly interactions between major powers have affected the development of new international relations. A deep learning network model is presented for this purpose. The deep learning model was used to identify the emotions of the survey results, analyze each person's emotional tendencies, and summarize and compare the data. Relevant questionnaire surveys were conducted using the online questionnaire survey method on individuals in various countries. The survey results in this paper demonstrate that 96.5 percent of Chinese, 89.3 percent of Russians, and 81.6 percent of Americans support friendly relations between major nations. Only a very small percentage of the investigators supported hostile relations, with their support being 1.06 percent, 3.11 percent, and 2.94 percent, respectively. Therefore, creating a win-win partnership between major powers is exactly what the people of all nations are calling for. In contrast to the past, it is no longer hostile and violent. People anticipate that more great powers will coexist peacefully.

## 1. Introduction

The course of world history demonstrates that the relationships between major powers have an impact on not only how the international community develops but also how the world is currently organized. Major nations are at the centre of the global stage as the world experiences a major change that is unprecedented. It is imperative to actively promote the creation of a global community of shared destiny as well as the idea and process of forging new international relations in light of the crucial question of how global relations will develop. In addition to being a crucial step in creating a world community with a shared future, the development of new international relations represents a significant advancement of the field. In the process of actively fostering the development of new international relations, it is important to highlight the regular international exchanges between major powers, which are based on reciprocal coordination and friendly interaction between nations, rather than competitive hostility. Additionally, maintaining international peace and stability depends heavily on the orderly expansion of trade between nations. Studying the friendly relations between great powers and creating a suitable new type of international relations are therefore crucial in the current international environment.

The article "Big Data Analysis of Benign Interaction of Great Power Relations and New International Relations Based on Deep Learning" was retracted in 2023. Reasons: signs of a paper mill; suspected computer-generated content; unreliable results or conclusions; lack of ethics approval or compliance.

International relations have always been a hot topic, and many scholars have made a series of related researches on it. Willardson and Johnson conducted research on arms transfer, organized and analyzed its related literature, and discussed the general adaptability between arms transfer and international relations theory. Starting from seven theories such as realism, liberalism, and constructivism, seven hypotheses were verified, and the results showed that the support for the realism hypothesis was limited [1]. Shih explored several illustrative practices of the Confucian typology of international friendly relations. According to the asymmetry of the strength and ability of the previous relationship, it is divided into four kinds of friendship, including Russia, North Korea, and Vietnam, aiming to maintain or even strengthen the Confucian ethical order, emphasizing the relevance of previous relationships that are considered to constitute friendship [2]. Etkin and Evcan attempted to understand and explain the changes in “why” and “how” and believed that it can reveal images more clearly. They also proposed reasons for understanding the multiple meanings of these changes and concepts, which require a special understanding of change [3]. This was done in order to understand and explain the various definitions and meanings of various concepts in international relations and other social research fields. The opportunity will be lost if reflection, foresight, and necessary revisions are not made, according to Suttner R who examined the changes and continuation of South Africa's foreign policy and identified the causes of its deteriorating global and regional status as well as the resurgence of South Africa's capacity to establish norms and agendas. Numerous academics use various research techniques when studying international relations. In this paper, a deep learning model is presented for research and analysis on the peaceful coexistence of superpowers and the contemporary form of international relations.

Deep learning is emerging machine learning technology, which is introduced into machine learning to make machines go further to artificial intelligence [4]. In recent years, research works related to deep learning have emerged in an endless stream. Some scholars brought the concept of deep learning to hyperspectral analysis and validated the qualification of stacked autoencoders by following typical hyperspectral information-based feature classification methods. At the same time, they provided a novel deep learning framework to combine features and thus could achieve higher analysis accuracy. Practice has also proved that it opens up a new window for further in-depth research, while also demonstrating the great potential of using deep learning techniques for more accurate hyperspectral data analysis [5]. Based on a deep learning architecture, Kermany et al. had developed a diagnostic tool to screen for all treatable blinding retinopathy and provided a clearer and more interpretable diagnosis by highlighting the areas identified by the neural network. Widespread application of artificial intelligence system in childhood pneumonia was confirmed [6]. Oshea and Hoydis introduced and discussed some new physical-level deep learning applications and proposed a fundamentally new approach to understanding the communication system as an autoencoder and showed how to extend this idea to networks of multiple transmitters and receivers and presented the concept of a radio transformer network. Experimental results show that the classification accuracy of deep learning based on convolutional neural networks is more competitive compared to traditional schemes relying on expert features [7]. Tom et al. introduced some important deep learning models and algorithms in many NLP and gave the process of their evolution, summarized and compared different models, and compared the past, present, and future of NLP [8].

The article "Big Data Analysis of Benign Interaction of Great Power Relations and New International Relations Based on Deep Learning" was retracted in 2023. Reasons: signs of a paper mill; suspected computer-generated content; unreliable results or conclusions; lack of ethics approval or compliance.

In this paper, a deep learning model is introduced in the analysis of the benign interaction of major power relations and the construction of new international relations. The opinions and views of the people of various countries on the relationship between major countries were collected through an online questionnaire. Through the built deep learning model [9,10] for emotion recognition, it is summarized into five viewpoints, namely, friendly relationship, alliance relationship, general relationship, no relationship, and hostile relationship. The experimental data shows that the people of China, Russia, and the United States support friendly relations between major powers by 96.5%, 89.3%, and 81.6%, respectively. Meanwhile the supporters of hostile relations only accounted for a very small number of investigators, and their support for hostile relations was 1.06%, 3.11%, and 2.94%, respectively. It is shown that most people maintain a friendly attitude towards the relations between major countries. Therefore, the new international relations should advocate the new concept of mutual help and win-win cooperation, establish a new concept of interests and destiny, and further maintain and develop the benign interaction between major powers.

The article "Big Data Analysis of Benign Interaction of Great Power Relations and New International Relations Based on Deep Learning" was retracted in 2023. Reasons: signs of a paper mill; suspected computer-generated content; unreliable results or conclusions; lack of ethics approval or compliance.

## 2. Construction of a New Type of International Relations

### 2.1. New Types of International Relations

#### 2.1.1. Definition

The concept of “win-win cooperation” is essential to developing a new type of international relations. In contrast to the old “zero-sum” game mentality, where you lose and I win, and you lose and I gain, “cooperation” and “win-win” refer to a relationship of mutual benefit. The path to achieving “win-win” is through the new form of international relations. “Win-win” and “cooperation” go hand in hand and are mutually beneficial.

#### 2.1.2. Meaning

Win-win outcomes are desired, and cooperation is the way to achieve them. A great power's growth is necessary to preserve international harmony and advance global economic growth, and a great power's growth and strength are favourable to international harmony and stability. The world experienced financial turmoil in 2008, and the economy as a whole experienced a Waterloo. The United States, Europe, and Japan, the three major western economies, all experienced a recession at the same time. It is well known that China, an emerging economy, has been crucial to the recovery of the world economy.

In the modern era, “win-win cooperation” is a crucial component of international relations theory. The main goal of international exchanges among the major powers is to establish win-win cooperation, which is consistent with the trend of economic globalization and democratization of international relations. It has a beneficial and extensive impact on the development and evolution of future international relations, opening up a new avenue for resolving intercountry conflict. The key concept in today's international relations is “win-win cooperation,” which is also the path to peace and prosperity.

#### 2.1.3. The Background Formed

*(1) Historical Perspective.* From a historical perspective, international relations are constantly changing and require the right guidance. After a large-scale war in Europe in the first half of the 17th century, the basic norms of modern international relations appeared. The Peace of Westphalia established at that time was a norm for international relations based on sovereign equality. Since then, many international treaties have been signed internationally, including the Vienna System, the Washington System, the Yalta System, the League of Nations, and the United Nations that has continued to this day. The United Nations Charter laid the foundation for modern international relations, but the confrontation between the two major military alliances led by the United States and the Soviet Union played an important role in international relations after World War II, leading to the Cold War that lasted for fifty years [11].

The article "Big Data Analysis of Benign Interaction of Great Power Relations and New International Relations Based on Deep Learning" was retracted in 2023. Reasons: signs of a paper mill; suspected computer-generated content; unreliable results or conclusions; lack of ethics approval or compliance.

After the Cold War, the Soviet Union in Europe died along with the Warsaw Pact, while NATO continued to develop and expand its legitimacy. In Asia, the United States still maintains a system of military alliances and strives to use it as the “cornerstone” of the East Asian region, strengthening and expanding its means. In order to prove its existence, the United States and its allies have resorted to any means to find or create “strategic opponents,” which has brought great harm to the stable development and peace of the Asia-Pacific region. Recently, issues such as the Ukraine crisis and the “rebalancing” of the US in the Asia-Pacific region have been filled with Cold War mentality. A military alliance built on the basis of an enemy is very different from its closedness, uniqueness, and peaceful development. Recently, issues such as the Ukraine crisis and the “rebalancing” of the US in the Asia-Pacific have been filled with Cold War mentality. A military alliance built on the basis of an enemy is very different from its closedness, uniqueness and peaceful development.

70 years later, the beautiful blueprint depicted in the UN Charter has not yet been completed [12], and local conflicts and group politics have not ended. The “new international relationship” centered on cooperation and win-win situation has just become a new relationship that conforms to the trend of the times.

*(2) International Perspective.* In an international perspective, the world expects major powers to play a more important role. Every major country is one of the largest economies in the world, and their words and deeds are under the spotlight. The interests of major powers have been closely integrated with global interests. Whether it is to promote economic development, to resolve various crises and contradictions, or to establish a fair and reasonable new world order, the participation of major powers is required [13]. This shows that all countries in the world are expecting great powers to play a greater role. In this process, the whole world has paid more and more attention to the responsibilities of major powers. This is a good opportunity for major powers to show their strength.

### 2.2. Positive Interactions between Major Powers

The development of a new kind of international relations benefits from the peaceful interaction between major powers. These nations with strong global influence and overall strength are the major factors currently influencing the global pattern. In the modern world, China, the United States, Russia, and Europe all play significant roles. The mutual cooperation between major powers must be taken into consideration when constructing a new type of international relations. Instead of ruthless competition, this new kind of relationship is based on coordination and cooperation between major powers as well as positive mutual influence.

The article "Big Data Analysis of Benign Interaction of Great Power Relations and New International Relations Based on Deep Learning" was retracted in 2023. Reasons: signs of a paper mill; suspected computer-generated content; unreliable results or conclusions; lack of ethics approval or compliance.

The meaning of positive interaction is as follows.

#### 2.2.1. Guide the Triangular Relationship between China, the United States, and Russia to Develop in a Nonconfrontational Direction

The trilateral relationship between China, the United States, and Russia has once again emerged as one of the major factors affecting global development in the world's most intense geopolitical competition today. For the time being, the United States views China and Russia as strategic rivals. China and the United States now engage in a much more intense strategic rivalry. Russia is playing a more competitive game with the US, Europe, and China, and the level of strategic cooperation between the two countries has significantly increased. The relationship between the United States and Russia will be challenging to improve in a short period of time due to the political opposition of the United States and the significant conflicts of geopolitical and strategic interests of the two countries, even though both the Presidents of the United States and Russia hope that it can [14]. While this is happening, there has been a year-long economic and trade dispute between China and the US. Many people are concerned that this will cause the Sino-US relationship to further deteriorate, which would be bad for both the US and the rest of the world.

As permanent members of the UN Security Council, China, the US, and Russia are all represented. International affairs would find it challenging to find a solution without their combined efforts. The trilateral relationship between China, the United States, and Russia should be pushed to a goal that is conducive to the realization of a community with a shared future for humanity by countries using their growing influence and international strategizing abilities.

#### 2.2.2. Build a Framework for Major-Country Relations with Overall Stability and Balanced Development

Russia and China are both global superpowers, and the two nations are situated close to one another. The two countries' interests share a lot of similarities. For instance, the smooth development of relations between China and Russia is a model for the relationship between major countries today in terms of military cooperation in acting and diplomatic trade. China and Russia steadfastly support and defend one another's development and core interests. There is now a comprehensive strategic cooperative partnership between China and Russia. The two sides adhere to the pragmatic cooperation of “nonalignment, nonconfrontation, and nontargeting of third parties” as the foundation of their strategic partnership, which is built on the basis of their respective development needs. Given that the world is presently experiencing its most turbulent period in a century, with frequent occurrences of uncertainty, “black swans,” and “grey rhinos,” Sino-Russian relations are the aspect of current international relations which is the most stable.

The article "Big Data Analysis of Benign Interaction of Great Power Relations and New International Relations Based on Deep Learning" was retracted in 2023. Reasons: signs of a paper mill; suspected computer-generated content; unreliable results or conclusions; lack of ethics approval or compliance.

The direction in which the relationship between China and the United States is moving merits attention. If China and the United States can work well together, they will undoubtedly play a key role in maintaining global stability and advancing global peace and development. China and the United States can and should seek a new strategy that differs from the conflict and confrontation between major powers in the past in the context of today's globalization. Economic growth, counterterrorism, preventing the spread of weapons, fighting transnational crimes, and stopping the spread of the epidemic are all issues that China and the US have in common. In light of the new circumstances, China and the US should forgo the “zero-sum game” that has traditionally existed between traditional major powers, actively pursue consensus, and encourage Sino-US relations to be based on coordination, cooperation, and stability.

#### 2.2.3. Promoting Major Powers to Strengthen Cooperation on Global Governance Issues

The global system is changing in light of the new historical circumstances. As a result, global governance is facing a number of fresh issues and difficulties [15]. Expanding the representation and voice of developing countries is a primary objective of the major powers in the reform of the international governance system in order to achieve a more equitable and sensible global order. The solution to global governance issues lies in enhancing international coordination and cooperation. The five permanent members should, first and foremost, improve coordination and cooperation to prevent conflicts between major powers that would have an impact on international governance. When developing new international regulations for areas like networks, deep seas, polar regions, air, and space, in particular, nations should work more responsibly together [16]. The second is to accurately grasp the UN's place in the world, actively promote the UN's proposed 2030 sustainable development goals, and actively engage with major world problems like climate change. The third step entails encouraging the G20 to take a more active role in society as a whole. It is essential to fully incorporate the new idea of international relations and promote nations' cooperation for their own interests in the process of global governance.

The article "Big Data Analysis of Benign Interaction of Great Power Relations and New International Relations Based on Deep Learning" was retracted in 2023. Reasons: signs of a paper mill; suspected computer-generated content; unreliable results or conclusions; lack of ethics approval or compliance.

### 2.3. Deep Learning

Although the concept of deep learning [17] is very short as it has been since its birth, the research on algorithm models has made great progress. Most of them are improved based on algorithms such as restricted Boltzmann machine (RBM) and automatic exposure (AE) algorithm.

Compared with the cultivation of advanced thinking, deep learning is to improve its ability to solve various complex and changeable problems by itself. Its specific performance is as follows: the ability to respond to thinking problems, the ability to judge complex things, the ability to further accurately understand problems, and so forth. The connotations of cognitive goals are shown in Table 1.

#### 2.3.1. RBM Algorithm

*(1) Algorithm Principle.* RBM is a unique structure of Markov random field [18]. It consists of a hidden layer *h* and a visible layer *v*. The difference from the common Boltzmann machine is that the weight connection in RBM only appears between layers, and the units within the layer are not connected, as shown in Figure 1.

The basis of the RBM model is statistical mechanics. Based on the energy probability model, when the parameter is a fixed value, RBM is the distribution of energy functions related to layer units *v* and *y*.

(1) $$\begin{array}{c} P\left(y\right)=\frac{e^{-E\left(v,h|\alpha \right)}}{S}. \end{array}$$

Formula (1) is an estimation expression for the RBM state, which is only valid for the two-layer structure composed of the visible layer and the hidden layer, where the *S* value normalizes the convergence factor, and its double accumulation formula is as follows:

(2) $$\begin{array}{c} S=\sum \left(v\right)\sum \left(h\right)e-\sum \left(y\right). \end{array}$$

For the RBM model of the double-layer structure, it can be expressed by a Bernoulli energy formula. The energy formula expression of the RBM model is

(3) $$\begin{array}{c} E\left(v,h|\alpha \right)=-A-B-C,\\ A=\sum_{j=1}^{m}b_{j}v_{j},\\ B=\sum_{i=1}^{n}c_{i}h_{i},\\ C=\sum_{i=1}^{n}\sum_{j=1}^{m}q_{ij}v_{j}h_{i}. \end{array}$$

In the above formula, *n* and *m* represent the unit datasets of visible layer and hidden layer, respectively; *q*_*ij*_ is the weight of the connecting edge between the visible layer and the hidden layer.

The article "Big Data Analysis of Benign Interaction of Great Power Relations and New International Relations Based on Deep Learning" was retracted in 2023. Reasons: signs of a paper mill; suspected computer-generated content; unreliable results or conclusions; lack of ethics approval or compliance.

When *v*_*j*_ follows a certain distribution probability, according to the RBM model, the independent active state parameters of the visible unit *v*_*j*_ and the hidden layer unit are obtained, and then the visible layer and the hidden layer can use Formula (4) to express their unit conditional probability:

(4) $$\begin{array}{c} P\left(h_{i}=1|v;\alpha \right)=\beta \left(\sum_{i=1}^{i}q_{ij}v_{j}+b_{j}\right),\\ P\left(v_{j}=1|h;\alpha \right)=\beta \left(\sum_{i=1}^{i}q_{ij}h_{i}+c_{i}\right). \end{array}$$

From the above formula, *β*(*y*) is the Sigmoid threshold function whose expression is

(5) $$\begin{array}{c} \beta \left(y\right)=\frac{1}{\left(1+e^{-y}\right)}. \end{array}$$

This expression is only valid for the two-layer structure consisting of visible layer and hidden layer. When the model structure is larger than two layers, the expression will be invalid. For the multilayer structure model with more than two layers, the Gaussian Bernoulli formula is generally used, and its formula expression is

(6) $$\begin{array}{c} E\left(v,h|\alpha \right)=-\frac{1}{2}D-B-C,\\ D=\sum_{j=1}^{m}{\left(v_{j}-b_{j}\right)}^{2}. \end{array}$$

The expression for the conditional probability distribution of continuous actual numerical RBM is

(7) $$\begin{array}{c} P\left(h_{i}=1|v;\alpha \right)=\beta \left(\sum_{i=1}^{i}q_{ij}v_{j}+b_{j}\right), \end{array}$$

(8) $$\begin{array}{c} P\left(v_{j}=1|h;\alpha \right)=I\left(\sum_{i=1}^{i}q_{ij}h_{j}+c_{i},1\right), \end{array}$$

In the above formula, 1 is the variance; *v*_*j*_ is continuous actual value; *Q*_*ij*_*h*_*i*_ indicates obeying the mean.

*(2) Deep Model.* Through Formulas (1)∼(4), the simplest two-layer structure deep network model of RBM can be established, and then data training is performed. The objects of Formulas (5)∼(8) are multilayer deep networks, which are trained on continuous real values. In other words, the simple overlapping of RBM networks constitutes a multilayer deep structure [19]. Deeper training model's visible layers are represented by the training results of simple RBM network model data. The result is used as the actual training data to solve the problem of continuous value data in practical applications. The deep network model is shown in Figure 2.

#### 2.3.2. AE Algorithm

*(1) Principle of AE Algorithm.* From a structural point of view, autoencoding is to encode the initial data of the visual layer. That is, a space set contains feature map data extracted from very complex input layer data, and these feature map data will be aggregated into hidden layers and output. The process of decoding is that the data space accepts the reflected feature map data [20] and reestablishes the data of the hidden output layer, so that the initial input data is roughly the same as the reconstructed data. The expression of the AE algorithm is

(9) $$\begin{array}{c} J\left(\varepsilon ,\varepsilon^{\prime }\right)=R+U,\\ R=\frac{1}{n}\sum_{j=1}^{n}L\left(x^{j},y^{j}\right),\\ U=\frac{\beta }{2}\left({\left\|\varepsilon \right\|}^{2}+{\left\|\varepsilon \prime \right\|}^{2}\right). \end{array}$$

In the above formula, *R* indicates that the model minimizes the reconstruction error; *U* is weight decay term; *ε* is output representation with respect to {*Q*, *b*} construction parameters; *ε*′ indicates that the output representation obtained after encoding is about {*Q′*, *b′*} construction parameters; *n* is sample data; *x* is original input dimension; *y* is reconstruction dimension.

*(2) Deep Structure Based on AE Algorithm.* Compared with RBM, the AE algorithm has a simpler structure and has a better effect on deep stacking to form a deep network structure. The training steps of the model are as follows: first, input the initial data into it, and encode the input data with the encoder. Then the decoder performs decoding and adjusts the relevant parameters of the encoder and the decoder to minimize the error of the reconstructed data, thereby obtaining the first layer of coding. Then, take the obtained first layer encoding as input data, and repeat the encoding process. It can be completed when all hidden layer data training is completed. When the top hidden layer is output, add a supervision layer. Finally, according to the added supervision layer standard, the hidden layer data is slightly adjusted, and the multilayer automatic encoding overlap can form the deep structure of the AE algorithm. Multilayer automatic coding is shown in Figure 3.

The article "Big Data Analysis of Benign Interaction of Great Power Relations and New International Relations Based on Deep Learning" was retracted in 2023. Reasons: signs of a paper mill; suspected computer-generated content; unreliable results or conclusions; lack of ethics approval or compliance.

## 3. Questionnaire Survey and Deconstruction of the New Type of Major Power Relations

This paper conducts a questionnaire survey on people from different countries among the three major world powers, China, Russia, and the United States. The content of the questionnaire survey is an opinion on what kind of relationship should be maintained between the major powers in the world at present. The survey results of the youth, middle-aged, and old age groups are summarized, respectively. The survey results are shown in the following table.

From Table 2, it can be seen that the relationship between major countries with the highest degree of support is friendly relations. The support levels of personnel from China, Russia, and the United States are 96.5%, 89.3%, and 81.6%, respectively. The supporters of hostile relations only accounted for a very small number of investigators, and their support for hostile relations was 1.06%, 3.11%, and 2.94%, respectively. It can be seen from the level of support of various countries that the building of a win-win cooperation between major powers corresponds to the appeal of the people of all countries and opposes the hostile and competitive relationship between the major powers in the past, organized into a data figure as shown in Figure 4.

The mentioned data is substituted into the multilevel deep structure training model as the initial data for training, so that the model can learn and improve continuously, and then the model is used to perform language recognition on the questionnaire responses of various countries. The recognition accuracy is shown in Table 3.

The average recognition accuracy of the depth recognition model based on the AE algorithm reaches 90%, while the average recognition accuracy of the depth recognition model based on the RBM algorithm is only 88%. The recognition accuracy of the deep recognition model based on the AE algorithm is relatively higher. Therefore, this paper selects the AE algorithm for further experimental investigation.

The deep recognition model based on the AE algorithm is applied to the network survey through the network to investigate the views of the people of various countries on the unreasonable relationship between China and the United States and between China and Russia and the relationship between Russia and the United States and use the deep learning model for identification. The results are shown in Figure 5.

From the data in Figure 5, it can be seen that the support rate of the Chinese people for the friendly relationship between China and Russia is 95.7%, and the support rate for the hostile relationship is only 1.77%. The Russian people's approval rate for Sino-Russian friendly relations is 91.4%, and the support rate for hostile relations is only 1.79%. It can be seen that the Chinese and Russian people hold an attitude of friendly coexistence and win-win cooperation towards Sino-Russian relations, which has been the key to the smooth cooperation between the two countries in recent years and the cornerstone of the common development of the two countries. Different age groups have roughly the same views on China and Russia. Many people hope that the two major powers of China and Russia will continue to maintain a friendly situation. Most of the supporters of the few hostile relations that appear are young people. They account for more than 90% of the supporters of hostile relations, because a small number of young people have a wrong view of Sino-Russian relations. At present, Sino-Russian relations are developing smoothly and are a model of major-country relations and neighboring relations.

The article "Big Data Analysis of Benign Interaction of Great Power Relations and New International Relations Based on Deep Learning" was retracted in 2023. Reasons: signs of a paper mill; suspected computer-generated content; unreliable results or conclusions; lack of ethics approval or compliance.

From Figure 6, it can be seen that there are still some differences in the current Sino-US relationship. The Chinese people's support rate for the friendly relationship between China and the United States is 63.5%, and the support rate for the hostile relationship has reached 22.4%. The American people's approval rate for Sino-US friendly relations is 41.6%, and the support rate for hostile relations reaches 31.9%. Most of the people who agree with hostile relationships are in the two age groups of 18–25 and 45–55. The reason for this phenomenon is the frictions and conflicts between China and the United States in the past, including the current economic and political frictions. Even so, most people of the two countries still hope that China and the United States live in harmony. The combination of China and the United States is a win-win situation. Conflict is a lose-lose situation. Cooperation is better than friction, and negotiation is better than confrontation. At present, there are some problems in Sino-US relations, but they are not in the interests of both sides. Although there are some differences between China and the United States, their interests are highly integrated and the scope of cooperation is extensive. Although there are some differences between China and the United States, their interests are highly integrated and the scope of cooperation is extensive. They should not be caught in the so-called conflict and confrontation but should promote each other and develop together.

The degree to which Americans and Russians support the various aspects of the bilateral relations is depicted in Figure 7. Only 40.5 percent of the Russian population supports a friendly relationship between Russia and the United States, while 84.1 percent of the population supports a hostile relationship. People of all ages in both Russia and the United States are pessimistic about the relationship between the two nations. In the United States, only 30.9 percent of people support a friendly relationship with Russia, while 79.9 percent support a hostile one. The two major powers, Russia and the United States, have frequently clashed in recent years. The relationship between Russia and the United States has once again reached a low point, particularly in light of the incident in Ukraine. There are still conflicts between the two nations. It is unlikely that relations between the United States and Russia will improve quickly due to political opposition in the United States and serious conflicts between the two countries' geopolitical and strategic interests, even though both the presidents of the United States and Russia express the wish that they can be improved.

The article "Big Data Analysis of Benign Interaction of Great Power Relations and New International Relations Based on Deep Learning" was retracted in 2023. Reasons: signs of a paper mill; suspected computer-generated content; unreliable results or conclusions; lack of ethics approval or compliance.

China, the United States, and Russia now have a different relationship than the Cold War's original three participants—China, the US, and the USSR. Russia and the United States will not be affected by China and Russia's close relationship. Russia-US relations are deteriorating for internal reasons. The improvement in Sino-US relations is unrelated to the decline in US-Russian relations. Russia and the United States are focused on political and military influence, China and Russia are focused on all-around cooperation, and Sino-US relations are centred on economy, trade, and global governance. However, there are also some interactions between China, the US, and Russia on a global scale. To encourage the development of constructive interactions in the trilateral relationship between China, the United States, and Russia and to advance the trilateral relationship between China, the United States, and Russia to a goal that is conducive to realizing a community with a shared future for mankind, each major country should utilize its growing influence and international strategizing capabilities.

## 4. Conclusion

This paper conducts a network survey based on a deep learning model in order to study how to construct a new type of major power relationship. The content of the survey is the views of people of various countries on the relationship between major countries, and the collected survey results are identified and analyzed by deep learning models to analyze their semantic sentiment trends and organize the data. The experimental data shows that although there are still conflicts and frictions between major powers, most people maintain a friendly attitude towards the relationship between major powers and support the friendly coexistence between major powers and win-win cooperation. Therefore, the construction of a new type of international relations should advocate a new concept of win-win, multiwin, and establish a new concept of new interests and destiny and implement a new approach of sharing responsibilities and emphasizing both righteousness and interests. Of course, there are still some flaws in the experimental investigation of this paper. Only the opinions of the people of China, the United States, and Russia are collected, and the opinions of people in other countries are not collected. There is a lack of universality and this needs to be improved and developed in future research.

## Figures and Tables

**Figure 1:** Restricted Boltzmann machine.

**Figure 2:** Depth model.

**Figure 3:** Multilayer autoencoding structure.

**Figure 4:** Questionnaire survey results.

The article "Big Data Analysis of Benign Interaction of Great Power Relations and New International Relations Based on Deep Learning" was retracted in 2023. Reasons: signs of a paper mill; suspected computer-generated content; unreliable results or conclusions; lack of ethics approval or compliance.

**Figure 5:** Different levels of support for Sino-Russian relations.

**Figure 6:** Different levels of support for Sino-US relations.

**Figure 7:** Different levels of support for Russia-US relations.

**Table 1:** Deep learning cognitive target connotation table.

Study type	Target level	Connotation
Shallow learning	Memory	Retrieve relevant information from long-term memory
	Understand	Constructing knowledge meaning from teaching information
Deep learning	Application	Apply acquired knowledge and skills in new situations
	Analyze	Clarify the relationship between the elements and their relationship with the whole
	Evaluation	Make value judgments on the knowledge and skills learned according to certain standards
	Create	Integrate elements into a coherent or functional whole

**Table 2:** The degree of support for relations between different major powers.

	Alliance (%)	Friendly relations (%)	General relationship (%)	No relationship (%)	Hostile relationship (%)
China	90.2	96.5	42.1	12.6	1.06
Russia	88.5	89.3	34.8	17.6	3.11
USA	79.6	81.6	56.9	13.5	2.94

**Table 3:** The recognition accuracy of the deep learning model.

	Alliance	Friendly relations	General relationship	No relationship	Hostile relationship
RBM	0.85	0.89	0.91	0.87	0.88
AE	0.91	0.93	0.90	0.88	0.88

## Data Availability

The data used to support the findings of this study are available from the corresponding author upon request.
